The article "Sickle Cell Disease in Children: Knowledge and Home-Based Management Strategies among Caregivers at a Tertiary Facility in Northern Ghana" was published in 2022. Journal: Biomed Res Int.

# Sickle Cell Disease in Children: Knowledge and Home-Based Management Strategies among Caregivers at a Tertiary Facility in Northern Ghana

**DOI:** 10.1155/2022/3384813

**Published:** 2022-07-07

**Authors:** Stephanie Ajinkpang, Oboshie Anim-Boamah, Kingsley Appiah Bimpong, Fatima Joyce Kanton, Joyce B. P. Pwavra, Alhassan Abdul-Mumin

**Affiliations:** ^1^Department of Pediatrics and Child Health, Tamale Teaching Hospital, Tamale, Ghana; ^2^School of Nursing and Midwifery, University of Ghana, Accra, Ghana; ^3^Department of Pediatrics and Child Health, School of Medicine, University for Development Studies, Tamale, Ghana

## Abstract

Sickle cell disease (SCD) is a serious genetic and inherited disorder. It has a physical, psychological, and socioeconomic impact on affected individuals including children and families. Globally, about 275,000 children are born annually with SCD, with an estimated 85% of these births being in Africa. In Ghana, an estimated 2% of infants that were screened were affected by SCD. Although extensive studies have been conducted on the burden on parents of children with SCD, little is known about how parents manage the disease among their children at home in our setting. This qualitative study explored the knowledge of caregivers of children with SCD, how they recognize/monitor complications of the disease and management strategies at home. An explorative qualitative study using the nonprobability purposive method was used to interview fourteen (14) caregivers of children with SCD who were recruited from the Tamale Teaching Hospital. In-depth interviews using an interview guide was used. A tape recorder was used to record each interview yielding a total of fourteen (14) audios. Audiotapes were transcribed verbatim. Data collected during these interviews were analyzed using inductive thematic content analysis. Caregivers have adequate knowledge of the signs and symptoms of SCD, its complications, and the various types their children have but fall short of knowledge on the cause of SCD. Knowledge acquired on SCD does not translate into caregivers' ability to effectively identify and monitor crises or complications at home. Home management strategies used by caregivers' were both pharmacological and nonpharmacological, and some used the combination to manage pain and monitor the health of their children. Even though the majority have used traditional medicine before, they prefer orthodox interventions which they consider more effective.

## 1. Introduction

Sickle cell disease (SCD) is a term that encompasses a series of inherited blood disorders, where there are abnormalities in the genes that codes the hemoglobin beta-subunit [1, 2]. In affected persons, there are two mutated globin genes, which are inherited from both parents [3]. The resultant abnormal hemoglobin has a tendency of polymerizing, leading to hemolytic anemia, vasoocclusive crises, and other features seen in the disease [1, 3]. This disease is often associated with negative family stigma and caregivers feeling a sense of blame for their children's condition [4].

SCD is the commonest hemoglobinopathy [5]. Globally, about 275,000 children are born annually with the condition, with an estimated 85% of these births being in Africa [6]. In sub-Saharan Africa, varied prevalence has been reported from screening programs. A screening program in Nigeria gave a prevalence of 3% [7], whereas a 1.19% prevalence was reported in Liberia [8]. An earlier screening program in Ghana noted that about 2% of infants that were screened were affected by the disease [9]. It has been shown that the global burden of SCD is increasing [10]. Grosse et al. estimated that in sub-Saharan Africa, early childhood mortalities from SCD-related complications ranged between 50% in places with good access to health care, and 90% in places where access to health care is limited [11].

SCD is a long-term condition characterized by an unimaginable level of recurrent pain and reduction in health-related quality of life [12, 13]. Although SCD carries this significant morbidity, gaps in the level of knowledge of this condition and its home-based care management practices have been reported among caregivers of children with the condition [14, 15], and this has significantly been associated with the occurrence of complications and negative well-being in affected children [15, 16]. In persons with SCD, comprehensive care involving nonmedical and medical strategies as well as self-management strategies is required [17]. Appropriate home-based measures include folic acid supplementation, penicillin prophylaxis, and adequate hydration [18, 19]. Inadequate caregivers' level of knowledge of SCD and the nonadherence to appropriate home-based care practices have been associated with the occurrence of SCD-related complications [15].

In the management of chronic diseases like SCD, coordination of activities related to the management of the disease is advocated for among caregivers and affected children, and it has been noted that tasks related to treatment compliance, such as recall of appointments and medications, are likely to be executed by parents [20].

This study sought to explore the knowledge of caregivers on SCD so that gaps if any could be identified for proportionate interventions to be instituted. This would help doctors and nurses attending to caregivers at our facility and beyond to increase awareness of the disease. Also, findings from this study would help in planning educative sessions for parents of children with SCD, to facilitate early diagnosis of crises and prevention of complications. Specific guidelines and protocols for patients with SCD may be established. This study will also help the nursing educational institutions to tailor their curriculum to close gaps identified in the home management of SCD.

## 2. Methodology

### 2.1. Study Design and Area

An exploratory qualitative design was employed for this study. This study design helped to obtain new information, insight, and awareness and to determine new patterns between the knowledge and management of sickle cell crises at home. It also promoted a better understanding of the variables under study. The Department of Pediatrics and Child Health of the Tamale Teaching hospital was the study site for the study. The facility serves as the only referral center for the five (5) regions in northern Ghana and parts of the Bono-East and Oti Regions. It also serves as a clinical training site for undergraduate medical and nursing students of the University for Development Studies, as well as multiple post-graduate health training colleges. The department manages patients with SCD in crisis at the children's emergency ward and the main children's ward and also runs a weekly SCD follow-up clinic supervised by a Pediatrician.

### 2.2. Study Population

The population for this study was caregivers of children with SCD who are on admission or were attending review at the sickle cell specialist clinic of the Tamale Teaching Hospital.

### 2.3. Inclusion Criteria

Caregivers (mothers and fathers) with children between the ages of 2 and 14 years were diagnosed with hemoglobin SS and SC and were willing to participate in the study. This age bracket was used because the youngest and oldest children enrolled in our SCD clinic are aged 2 and 14 years, respectively.

### 2.4. Exclusion Criteria

The exclusion criteria is caregivers of children with SCD who were not willing to participate in the study.

### 2.5. Sampling

Purposive sampling was employed to select the participants for the study. This sampling was used to enable us to select a sample based on the experiences of the participants allowing for the selection of information-rich cases which serves to yield insights and an in-depth understanding of participants' experiences. Saturation was reached when about 14 participants were interviewed. Saturation is said to have reached when the researcher gathers data to the point of diminishing returns when nothing new is being added [21].

### 2.6. Data Collection Procedure and Tool

In-depth interviews using an interview guide was employed. The first author conducted the interviews in Dagbanli (the predominant local language in the Northern Region of Ghana) and English. Caregivers who presented their children for review or those on admission were approached for participation in the research. Those who were willing to participate were provided with written consent in English language and translated into a language they understood to complete.

Interviews were done in a quiet room in the hospital at the convenience of participants to ensure participants' anonymity and privacy, and some were done at the homes of the participants. The interview lasted for about 50 to 60 minutes and in a language they understood. Detailed field notes of the environment, nonverbal cues, interruptions, and personal reflections about observations made during the interviews were kept. Interviews in Dagbani were translated and transcribed into the English language verbatim. After the interview, participants were acknowledged and asked if they could be contacted after the interview for further clarification or verification of their responses in the course of the study. All interviews were audiotaped.

### 2.7. Data Analysis

Thematic content analysis (TCA) was employed for analyzing the data. This involves a descriptive presentation of qualitative data. This method involves looking across all the data to identify the main themes that summarize all the views collected [22]. In our study, this was done by placing major ideas into codes, which were later reorganized into themes, that summarized the ideas of the participants interviewed.

### 2.8. Ethical Considerations

Ethical clearance for this study was obtained from the Ethics and Research Review Board of the Christian Health Association of Ghana (CHAG) with reference number CHAG-IRB10022019. Permission was also obtained from the research department of the Tamale Teaching Hospital. Written informed consent was obtained from all caregivers before they were enrolled in the study, and they were assured that their responses would be anonymous. No participant identifiers were collected.

## 3. Results

### 3.1. Background Characteristics of Caregivers'

The majority (9, 64.3%) of the caregivers interviewed were mothers, and the age range of 20-39 years had the most participants (6, 42.8%). All caregivers interviewed were married. Tertiary level education was attained by majority (8, 57.1%) of the caregivers, and half of them were civil servants. The genotype SS was the most common (9, 64.2) among the children of the caregivers in our study.  Table 1 gives the baseline characteristics of the caregivers in our study.

### 3.2. Caregiver's Knowledge of SCD in Children

Participants were asked if they know anything about SCD. Four subthemes were generated from the data on this objective. They identified pain, fever, and yellowish eye or urine as some signs that could be exhibited by the children. This study identified a gap in knowledge where caregivers were unaware of the cause of SCD and its complications yet are aware of the signs and symptoms and various types their child or children were diagnosed with.

The subtheme of etiology described participants' knowledge about the etiology of SCD. This study identified a gap in knowledge where caregivers were unaware of the cause of SCD. Only two participants were able to mention that the disease is inherited as illustrated by these quotes:

“I think it is not an infectious disease whereby you easily trap it, you get that through your parents. It's hereditary something. If your parents have it you're likely to also get it” by participant 6 and “….for my little knowledge as we have been coming for the clinic we were told its genetic because it's from father to child or mother to child. So that's the only way you can get sickle cell. Its blood related.” (participant 12)

Other caregivers erroneously attribute SCD to other local misfortune:

“Some people say disease or ‘zunzuya' (worms) they cause it or whatever. So the worms if the children don't eat the worms will get strength and eat inside their stomach but when they eat they (worms) become weak. If you eat that they become weak, but if you don't eat they become stronger isn't it? It's all about your food.” (participant 5)

Another participant added that:

“What I know is that it's like when you are some type and you marry another type….I do not know but I think it's something to do with the man and the woman. I don't know if it's the blood type or what. It's like if one is positive and the other is negative.” (participant 13)

Despite the gap in the etiology of SCD, caregivers knew some of the signs and symptoms of the disease. Caregivers identified pain, fever, swelling of the limbs, difficulty in breathing, yellowish eyes, and urine as some of the signs and symptoms of SCD.

This is corroborated by the following extracts from the transcript.

“Sometimes I will see their hands swollen and sometimes they will say my hand is paining me, my backbone, mama press my here, press my here. The boy sometimes the back and the chest he can't breathe” (participant 4); “temperature rising, he too sometimes he coughs, he says he experiences pain but because he is a child I don't know if it true or not especially his joints” (participant 9); “the first signs are jaundice, pains especially joint pains, they have some temperature especially when they have infection or malaria.” (participant 12)

Awareness of complications is vital in understanding the severity of the disease. Although signs and symptoms were well identified, complications that could arise from the disease were not well known. Nonetheless, few (2) caregivers were able to identify anemia and infection as complications of the disease. A caregiver illustrated that “they are too stressed, they are too tired but I don't know if it's because of the disease. They easily get tired.” (participant 1), and other caregiver illustrated that “some complications are anemia and infections.” (participant 6)

Regarding knowledge of the type of SCD of their children, all but two (2) of the caregivers were aware of the types their children or child are suffering from. These caregivers were completely unaware of the SCD type of her child, which was illustrated as “…eeemm, for as in the local language they say ‘Darimihi' but they did not tell me the type of SCD the child had” (by participant 8) and “it's like A or is it B or something like.” (by participant 5)

### 3.3. Prevention of Crises and Home-Based Management

Several preventive management strategies were employed by caregivers. Aside from the hospital care and management, caregivers do indulge in home care to keep their children healthy and manage complications and crisis. Caregivers ensured that the children took enough water, avoided mosquito bites, and took healthy food that prevented anemia. Protection from infection and reduced exposure to extremes of weather were other strategies employed.

With regard to hydration, some caregivers illustrated: “We take precaution that you told us to do, let them take a lot of water” (participant 1), “he drinks a lot of water” (participant 11), and “as for water they take a lot, especially this dry season. The two of them alone can take a bag of water in a day.” (participant 12)

In addition, some caregivers prevented their children from exposure to cold weather as illustrated as

“Mostly even this time if he is going to sleep, I wear him pullover with long trouser, bath him with warm water.” (participant 7)

Just a few (2) made mention of preventing the child from extreme heat:

“And I learnt also that they don't want too much heat so that is also there.” (participant 1)

“They said they are very delicate, she shouldn't be exposed to the hot sun and she shouldn't be exposed to cold.” (participant 13)

Aside taking enough water and preventing extreme weather conditions, some caregivers take extra precautions to ensure that their children do not get malaria, which can be a precipitating factor for crises. This is illustrated by these two quotes: “I protect them from mosquito bites that's the first thing” (participant 2) and “that we should be very careful about malaria because they said if she gets malaria it will generate into a whole lot of problems.” (participant 13)

Some caregivers also elaborated on the kind of food they give their children. A lot of the participants indicated that they give the children normal family food and nothing different. A few indicated that they give them beans, eggs, leafy foods, as supported by the statement “Doctor said I should give them leafy foods such as aleefu as well as mixing with beans.” (participant 5)

Some pharmacological methods used by caregivers included the use of Penicillin V and Folic acid (routine drugs). Some caregivers illustrated: “he takes penicillin V and folic acid” (participant 14) and “as for drugs we have folic acid and penicillin V and vitamin C.” (participant 13)

Caregivers used different strategies to manage complications and crises. The major complications or crises they managed at home were pain and fever. They used pharmacological and nonpharmacological methods to manage pain as well as the fever. Some of the pharmacological strategies included the use of prescribed and over-the-counter drugs. Examples of such drugs included ibuprofen syrup/gel and paracetamol. The following extracts corroborated this finding: “I do sponge, is that the right term? Then if there is para syrup I give her” (participant 6), “for the fever I will give paracetamol and if I don't see changes I send him to the hospital” (participant 7), “at times I just give some paracetamol syrup and make sure I monitor especially when they have a temperature (high) and towel the body (tepid sponge). But if I see it is not subsiding I quickly rush them to the hospital” (participant 12), and “When the fever comes in the night we manage till daybreak then I will get Brufen” (participant 5).

The nonpharmacological methods employed by caregivers include massage with gels and placing warm towels on the affected part. This was supported by these quotes: “for pain, Oohh I use mentholated ointment to massage him”(participant 11); “so what we do is that we get hot water and small napkin inside and put on the part that is paining” (participant 13); and “when he is in pain I boil water and soak a towel in it to put on the legs to stop the pain but it wasn't going.” (participant 8)

## 4. Discussion

This qualitative study explored the knowledge of caregivers of children with SCD, their ability to prevent crises at home, as well as exploring some management techniques employed at home to manage crisis and ensure the wellbeing of these children. Knowledge of the type of SCD and signs and symptoms were adequate; however, knowledge regarding the etiology of SCD as well as the complications were of concern. Concerning the prevention of crises and home-based management strategies, caregivers ensured that the children took enough water, avoided mosquito bites, and took healthy food that prevented anemia. Protection from infection and reduced exposure to extremes of weather were other strategies employed. Pharmacological and nonpharmacological methods employed included the use of penicillin V and Folic acid, massaging affected parts with gels, and placing warm towels on these places.

The study identified that a majority of caregivers were aware of the various types of SCD that their children were suffering from as well as the on signs and complications of the disease. However, knowledge on the cause of SCD was lacking. This finding is similar to a study by Van Niekerk in South Africa where it was seen that majority of caregivers had some knowledge of the disease [23] but their knowledge regarding the cause was inadequate. Most of the caregivers either had no idea of the cause or attribute the disease to local beliefs and supernatural elements as participant 5 stated that “Some people say disease or ‘zunzuya' (worms) they cause it or whatever. So the worms if the children don't eat the worms will get strength and eat inside their stomach but when they eat the (worms) become weak. If you eat that they become weak, but if you don't eat they become stronger isn't it? It's all about your food……” This finding is similar to a study by Van Niekerk who also noted that a number of caregivers interviewed did not know the exact cause of SCD [23]. The attribution of the etiology to local beliefs and supernatural elements was not surprising as other studies in Ghana have reported the disease to supernatural causes [24, 25]. This is a very disturbing finding.

Preventive programs such as genetic screening for SCD or carrier state before marriage or pregnancy is one of the most effective means of reducing the burden of SCD [26]. Unfortunately, Ali and Razeq noted that caregivers of children with SCD in their study did not know their carrier status, until the first diagnosis of their children [27]. One reason for the inadequate knowledge on the cause of SCD could be the inadequacy of genetic counseling, which is intended to provide empirical information about genetics to help individuals understand the impact of a genetic diagnosis on their life and that of their children.

Compliance with recommended home-based measures such as folic acid supplementation, penicillin prophylaxis, hydration, and nonpharmacological measures such as maintaining normal body temperatures are some useful ways of managing the disease [18, 19]. Although SCD-related complications are to be managed in hospitals, home care and management strategies are key since the disease is unpredictable. Caregivers of children with SCD in this study used similar methods of managing crisis including pain management as it was one of the most frequent complications. Dampier et al. noted that with appropriate training, complications of SCD such as recurrent pain could be managed successfully at home [28].

These methods were classified as pharmacological and nonpharmacological. Pharmacological interventions were more common than nonpharmacological interventions with respondents reporting a preference for conventional medicines. The majority had used traditional medicines, but only a few were current users as traditional medicines were viewed as ineffective. The pharmacological methods involve the use of drugs at home to either manage complications or prevent them from occurring. Caregivers in this study give penicillin V and folic acid as part of their routine drugs from the hospital and paracetamol and ibuprofen syrup for pain and fever. Penicillin prophylaxis has been strongly recommended as a preventive measure in SCD management [19]. Home-based usage of analgesics is also common among patients with SCD [28].

The nonmedicinal method in this study included bathing children with warm water.

## 5. Conclusion, Limitations and Recommendations

Caregivers of children with SCD have adequate knowledge of the signs and symptoms of SCD, its complications, and the various types but fall short of the main and related cause of SCD. Knowledge acquired on SCD does not translate into caregivers' ability to effectively identify and monitor crises or complications at home. Physical examination such as splenic palpation was never mentioned, and measurements requiring the use of devices such as thermometers were limited among participants. The fact that some have older children with the disease, past personal experience was a major contributor to the effective monitoring of children at home by some few caregivers. These findings show that there is a need to remind/teach nurses the importance of physical assessment and educating the patients and caregivers.

This study has revealed that caregivers used pharmacological and nonpharmacological strategies or a combination of both strategies to manage and monitor the health of their children at home. Even though the majority have used traditional medicine before, they prefer orthodox interventions which they consider more effective.

The study team acknowledges the limitations of the study. The relatively small sample size and the specific context of the study were aimed at acquiring rich descriptive data. As a result, the sample may not be representative of the general population and generalization of the findings should be done with caution. However, the findings are consistent with other studies in Ghana and other African countries, and therefore transferability is possible when there is similarity in context.

We recommend that hospitals providing antenatal care (ANC) should provide education and genetic counseling to parents so that they have at least basic knowledge on the causes, signs and symptoms, and complication of management of SCD. Also, there is a need for a wider population level of premarital counselling and sickle cell genotyping to be done for would-be couples. Caregivers should adopt more than one home management strategies to effectively recognize and monitor crises or complications at home. In addition, a simple fact sheet explaining the condition, its cause, and inheritance should be given to all parents seen at the SCD clinic. Routine distribution thereof may be helpful in correcting misconceptions as well as providing something that can be easily shared with family or referred to in the future. The translation of this fact sheet into other languages, such as Dagbanli and other popular languages in northern Ghana, could further improve the reach of this fact sheet.

## Figures and Tables

**Table 1:** Background characteristics of caregivers'.

Baseline characteristic	Frequency (%)
Caregiver	
Mother	9 (64.3)
Father	5 (35.7)
Age of caregiver (years)	
<20	4 (28.6)
20-39	6 (42.8)
≥40	4 (28.6)
Marital status of caregiver	
Married	14(100)
Divorced	0
Educational level	
None	1 (7.1)
High school	5 (35.8)
Tertiary	8 (57.1)
Employment	
Civil servant	7 (50.0)
Trading	4 (28.6)
Unemployed	3 (21.4)
Genotype	
SC	5 (35.8)
SS	9 (64.2)
Number of children with SCD	
1	2 (14.3)
2-3	8 (57.1)
4 and above	4 (28.6)

## Data Availability

The dataset we used to support the findings of our study is available from the corresponding author on reasonable request.
